The article "Heart Rate Variability and Chronic Kidney Disease in Patients with Type 2 Diabetes" was retracted in 2023. Reasons: signs of a paper mill; compromised peer review; unreliable results or conclusions.

# Heart Rate Variability and Chronic Kidney Disease in Patients with Type 2 Diabetes

**DOI:** 10.1155/2022/2475750

**Published:** 2022-05-17

**Authors:** Wei Shi, Jing Zhang, Dan Chen, Xiaolei Chen, Wei Duan, Hongmei Zhang

**Affiliations:** ^1^Department of Endocrinology, Hubei Integrated Traditional Chinese and Western Medicine Hospital, Hubei University of Chinese Medicine, 430015 Wuhan, Hubei, China; ^2^Department of Endocrinology, Kunming First People's Hospital, Kunming Medical University, 650101 Kunming, Yunnan, China; ^3^Department of Endocrinology, The Central Hospital of Wuhan, Tongji Medical College, Huazhong University of Science and Technology, 430015 Wuhan, Hubei, China

## Abstract

To evaluate whether heart rate variability (HRV) as a measure of cardiac autonomic neuropathy (CAN) is associated with chronic kidney disease (CKD) in Chinese adults with type 2 diabetes mellitus (T2DM) in China. 392 individuals of T2DM were entered in this study, all these subjects undertook the Holter electrocardiogram for 24 hours to get the HRV parameters. Of these T2DM patients, 126 (37.3%) had CKD, and most of the HRV parameters were lower in this group than in those without CKD. Decreased HRV parameters were strongly related with CKD in Spearman's correlation analysis. After adjustments for variables, the logistic regression showed that standard deviation of the averaged normal RR intervals for all 5-minute segments (SDANN) was independently associated with decreased estimated glomerular filtration rate (eGFR < 60 mL/min/1.73 m^2^) (OR = 0.988; 95% CI, 0.978-0.998; *P* = 0.015) and increased urine albumin : creatinine ratio (UACR) ≥ 30 mg/g Cr (OR = 0.992; 95% CI, 0.985-0.998; *P* = 0.015). A decreased 24-hour time domain HRV parameter, SDANN, was strongly associated with both eGFR and UACR among Chinese T2DM.

## 1. Introduction

Type 2 diabetes mellitus (T2DM) associated chronic kidney disease (CKD) becomes the major contributor of end-stage renal disease and is strongly associated with cardiovascular events and death [1]. There has been evidence that in CKD, progression of renal failure continues despite tight and early control of glucose, blood pressure, and other traditional risk factors [2]. Thus, it is vital to look for better treatment options to reduce the incidence rate and fatality rate related to CKD.

Cardiac autonomic neuropathy (CAN) is often overlooked though it is known as a common complication of diabetes mellitus [3–5]. This disease is not only related to cardiovascular disease [6] but is also considered an important risk factor for CKD [1]. However, in clinical studies of CAN, diagnostic criteria, assessment methods, and demographics have varied, and the reported prevalence rates have been inconsistent [3–5]. It is considered that using 24-hour ambulatory electrocardiographic monitoring for analyses of heart rate variability (HRV) in the early stages of CAN is a sensitive way and does not cause inconvenience to the patients [7].

Although the relationship between CAN and renal dysfunction was discussed in several studies, the results had been inconsistent. As for the different characteristics of the researches, the races of most studies were Caucasians and the scales of these studies were small. Many of the researches had focused on patients of type 1 diabetes; the indices of CKD were different, such as glomerular filtration rate, albuminuria, or both; and the markers of CAN were also diverse and complicated [8–13]. Yet, Asian diabetic populations, including the Chinese, other than Caucasians, were showed to increase susceptibility to renal complications by consistent data [14].

This study focused on an association between HRV analyses including time and frequency domain parameters and two CKD markers (estimated glomerular filtration rate (eGFR) and albuminuria) in Chinese patients of T2DM

## 2. Subjects and Methods

### 2.1. Participants

This was a cross-sectional study that included 446 participants with T2DM in the inpatient department of Kunming First People's Hospital between February 2013 and April 2015. The including criterions were adults with T2DM, and all the participants had carried Holter monitoring for 24 hours. The excluding criterions were as follows: acute complications of T2DM, severe acute or chronic infection, dialysis or kidney transplantation, or any severe comorbidity affecting life expectancy. A total of 392 patients were finally analyzed.

Informed consent was signed by all the patients in our study. T2DM was diagnosed according to the Chinese Diabetes Society criteria [15]. CKD was assessed based on the levels of eGFR and urine albumin : creatinine ratio (UACR). The patients enrolled in our research were divided into subgroups according to eGFR and UACR (described below). All the enrolled patients were allowed to continue their previous treatment regimens for T2DM and hypertension. The Institutional Review Board of Kunming First People's Hospital approved the study protocol. The clinical trial registration code was obtained from the website of https://clinicaltrials.gov/(NCT02996539).

### 2.2. Clinical Examination and Laboratory Assays

A physician interviewed the medical history of the subjects including history of hypoglycemic episodes, drinking, and smoking habit and medication history. The anthropometric measurements were measured by a trained medical worker including the blood pressure, height, and weight of the subjects. The calculation formula for body mass index (BMI) was body weight, in kg, t divided by height in meters squared (kg/m^2^). A smoker was regarded as a subject smoking ≥ 1 cigarette per day, continuous or accumulated for 6 months. An alcohol drinker was defined as a subject consuming >20 g of alcohol per day in the past month. We defined the following conditions as hypertension: if the subject's systolic blood pressure ≥ 140 mmHg and/or diastolic blood pressure ≥ 90 mmHg, or the subject has history of taking antihypertensive drugs. Diabetic retinopathy (DR) was evaluated by an ophthalmologist.

Blood samples from all the subjects were collected after overnight fasting for 10 hours. Urine samples were collected for 24 hours. All these samples were analyzed at medical laboratory center of Kunming First People's Hospital. We used the urease-ultraviolet rate method to determine blood urea nitrogen (BUN) and picric acid method to analyze serum creatinine (SCr), respectively. An enzymatic colorimetric method was used to detect serum uric acid. Immunoturbidimetric analysis and enzymatic method were used to analyze urine albumin and creatinine, respectively. All these were analyzed by automatic biochemical analyzers (AU5403, AU5405, and AU5407, Olympus). High-performance liquid chromatography assay was used to analyze serum hemoglobin A1c (HbA1c) (H9, Pumen technical Corp., Shenzhen, China).

### 2.3. Assessment of CKD

CKD was diagnosed based on eGFR and albuminuria: the levels of eGFR less than 60 mL/min/1.73 m^2^ calculated by the modification of diet in renal disease (MDRD) equation in Chinese [16], or the levels of UACR greater than or equal to 30 mg/g [1]. Albuminuria was assessed by UACR which was measured from 24-hour urine samples that are collected. Patients were categorized as follows: low-eGFR (<60 mL/min/1.73 m^2^), high-eGFR (≥60 mL/min/1.73 m^2^) and UACR_1_ (normal albuminuria <30 mg/g Cr), UACR_2_ (30-299 mg/g Cr), or UACR_3_ (>300 mg/g Cr).

### 2.4. Assessment of HRV

A 3-channel digital Holter monitor (CB-2302-A, Zhongjian, Wuxi, Jiangsu, China) was used for all subjects for 24 hours to obtain the HRV measurements. A trained operator who was ignorant of the patients' clinical status reviewed and analyzed the data. QRS complex were detected and flagged by the specially designed software (CB Series ECG Regression Analysis System, Zhongjian, Wuxi, Jiangsu, China).

HRV analysis consists of time-derived and frequency-derived parameters. Regarding the time-derived, 4 indices were measured, each in milliseconds (ms): SDNN, standard deviation of the RR interval; SDANN, standard deviation of the averaged normal RR intervals for all 5-minute segments; SDNN index, the mean of the standard deviations of all normal RR intervals for all 5-minute segments; and RMSSD, the root mean square difference of successive RR intervals. The frequency-derived measures were as follows: low frequency (LF, >0.04 Hz and <0.15 Hz), high frequency (HF, >0.15 Hz and <0.4 Hz), and the ratio of low-to-high-frequency power (LF/HF). SDNN and LF/HF reflect the sympathovagal balance. SDANN, SDNN index, and LF reflect the activity of sympathetic nerve. RMSSD and HF reflect the activity of vagal nerve [17, 18].

### 2.5. Statistical Analysis

Our results are showed as mean ± standard deviation or median (25th-75th percentiles) for continuous variables and number (percentage) for categorical variables. Bivariate parameters between patients with relatively low or high eGFR were compared by Student's *t*-test or Mann–Whitney *U* test. Trivariate parameters among patients in different UACR groups were compared by ANOVA test or Kruskal-Wallis test. Categorical variables were compared using the chi-squared test. Spearman's test was used to assess univariate correlations between HRV parameters and different clinical characteristics. Binary logistic regression (for eGFR and UACR) was used to reveal the independent association between HRV and CKD. This included HRV parameters (described above) and the following potential risk factors as confounders: age, gender, BMI, duration of T2DM, drinking status, smoking status, hypertension, DR, the prevalence of hypoglycemia, HbA1c levels, and use of insulin, renin-angiotensin-aldosterone system (RAAS) inhibitor, diuretic, or beta-blocker. Statistical analysis were carried out in SPSS version 22.0 (SPSS, Chicago, IL, USA). A two-tailed *P* value below 0.05 was considered in a statistical sense.

## 3. Results

### 3.1. Population Characteristics

We finally analyzed 392 T2DM patients, 53.1% of them were women; the average age of the subjects was 59.1 ± 0.59 years; the mean diabetes duration was 5.99 ± 0.34 years; and the mean level of HbA1c was 8.8 ± 0.1%. The prevalence of CKD was 37.3% of the enrolled patients.

Baseline eGFR measurements were available for 384 patients. Of these, 13% (50/384) were in the low-eGFR group (Table 1). Patients in the low-eGFR group were significantly older, had a higher mean BMI, longer duration of T2DM, higher prevalence of hypertension and hypoglycemia compared with patients in the high-eGFR group; the low-eGFR group also had higher levels of BUN, SCr, uric acid, and UACR; a higher proportion of patients in the low-eGFR group were taking RAAS inhibitors and insulin. However, the two groups were statistically similar with regard to gender ratio, the status of drinking and smoking, prevalence of DR, HbA1c levels, and antihypertensive treatments except for RAAS inhibitors and oral antihyperglycemic drug.

Baseline UACR measurements were available for 344 patients. Of these, 61.6% (212/344) were considered to have normal UACR (UACR_1_), 29.7% (102/344) were in the higher UACR groups (UACR_2_ and UACR_3_), and 8.7% (30/344) were specifically in the UACR_3_ group (Table 1). Compared with patients in the UACR_1_ group, the following were much higher in both the UACR_2_ and UACR_3_ groups: BMI, duration of T2DM, the prevalence of DR, and use of RAAS inhibitors. The prevalence of hypoglycemia and HbA1c levels in the UACR_2_ group were significantly higher relative to the UACR_1_ group. The UACR_3_ group had a significantly greater proportion of hypertension and lower eGFR levels than the UACR_1_ group. The SCr, serum uric acid levels, and the proportion of taking diuretics for patients in the UACR_3_ group were significantly higher relative to either the UACR_1_ or UACR_2_ group. However, all the UACR groups were statistically similar in age, gender, smoking, drinking, BUN, use of calcium antagonists and beta-blockers, and treatments of diabetes.

### 3.2. Association between HRV and CKD (eGFR and UACR)

As compared with the high-eGFR group, the low-eGFR group had significantly less HRV (SDNN, *P* = 0.001; SDANN, *P* ≤ 0.001; SDNN index, *P* = 0.021; and LF/HF, *P* ≤ 0.001; Table 2).

The patients in the UACR_3_ group had lower HRV parameters relative to the UACR_1_ group, as shown by the following (Table 2): SDNN, *P* ≤ 0.001; RMSSD, *P* = 0.011; SDANN, *P* ≤ 0.001; SDNN index, *P* ≤ 0.001; LF, *P* = 0.001; and HF, *P* = 0.016. When compared with patients of the UACR_2_ group, the patients of the UACR_3_ group had lower levels of SDNN (*P* = 0.005), RMSSD (*P* = 0.032), SDANN (*P* = 0.005), SDNN index (*P* ≤ 0.001), and LF (*P* = 0.028). The patients of the UACR_2_ group only had lower levels of SDNN than these of the UACR_1_ group (*P* = 0.031).

The prevalence of CKD was negatively correlated with SDNN (*r* = −0.193, *P* ≤ 0.001), SDANN (*r* = −0.223, *P* ≤ 0.001), and SDNN index (*r* = −0.134, *P* = 0.014) in Spearman's correlation analysis (Table 3). In addition, UACR was negatively correlated with SDNN (*r* = −0.198, *P* ≤ 0.001), SDANN (*r* = −0.176, *P* = 0.001), SDNN index (*r* = −0.194, *P* ≤ 0.001), LF (*r* = −0.161, *P* = 0.003), and LF/HF (*r* = −0.111, *P* = 0.04), and eGFR was positively associated with LF/HF (*r* = 0.136, *P* = 0.008). We also found that age, BMI, diabetes duration, presence of DR, prevalence of hypoglycemia, HbA1c levels, smoking, drinking, and use of insulin, a RAAS inhibitor, diuretic, or beta-blocker were closely associated with HRV parameters.

Binary logistic regression analysis was performed to investigate an independent association between HRV and CKD (Table 4), with covariates for the gender, age, BMI, diabetes duration, drinking, smoking, presence of DR and hypertension, prevalence of hypoglycemia, HbA1c levels, and the use of insulin, an RAAS inhibitor, diuretic, or beta-blocker. We found reduced SDANN (*P* = 0.015), older age (*P* ≤ 0.001), and high levels of BMI (*P* = 0.011) were associated with increased risks for eGFR < 60 mL/min/1.73 m^2^. Low levels of SDANN (*P* = 0.015) and DR (*P* ≤ 0.001) were strongly associated with increased risks for albuminuria (UACR ≥ 30 mg/g Cr). This shows that reduced SDANN was independently associated with lower eGFR and higher UACR.

## 4. Discussion

The associations between CKD and 24-hour HRV parameters (time and frequency domains) among Chinese T2DM patients was explored in this study. It was found that most of the time and frequency domain HRV indices were less in both the low-eGFR group and higher UACR group (UACR_2_, UACR_3_) relative to the high-eGFR and UACR_1_ groups, respectively. Moreover, we found that SDANN was closely associated with both lower eGFR and higher UACR, the 2 important markers of CKD, and this relationship still established independently after adjusting for many common hazard factors, such as age, gender, BMI, diabetes duration, drinking status, smoking status, presence of hypertension and DR, prevalence of hypoglycemia, HbA1c levels, and use of insulin, RAAS inhibitors, diuretics, or beta-blockers. As the SDANN mainly reflects the imbalance of cardiac autonomic function and is related to increasing the activity of sympathetic nerve and decreasing the activity of vagal nerve, our results revealed that the sympathovagal imbalance was involved in CKD in Chinese patients of T2DM.

Although the similar association between CAN and CKD in diabetes after adjust for several risk factors was demonstrated in a few previous study [9, 10, 13], there are three different aspects between our study and the previous ones. Firstly, we use better anti-inference tools for CAN time and frequency analysis other than cardiovascular reflex tests [9, 10, 13]. Secondly, Yun et al. [9] and Eun Jun et al. [13] showed CAN was strongly associated with CKD evaluated by eGFR or UACR; in our study, we displayed CAN was related to both eGFR and UACR. Thirdly, unlike the previous study [9, 10, 13], we carried out the study in the Chinese T2DM population.

An earlier Chinese study, which had focused on the association between time domain 24-hour HRV parameters and albuminuria, had also shown that reduced SDANN, SDNN index, and SDNN were linked with albuminuria [19]. In our research, we found out independent associations between SDANN and eGFR and between SDANN and UACR. In contrast to a former study among white European and South Asian patients with T2DM [20], we found no association between HRV parameters related to parasympathetic activity (RMSSD and HF) and renal function. The differences in these results may be because of differences in the selection of patients and in methods of evaluating HRV. For example, the duration of T2DM is known to have an effect on CAN [21], and in the previous study, the duration of diabetes was more than 10 years; this is much longer than our study (the median duration of 4 years). Furthermore, the HRV parameters in the past studies were recorded for the short term with respiratory adjustment, while we recorded HRV for 24 hours.

The underlying mechanisms by which CAN may contribute to the progression of CKD has been reported in previous studies [12, 18, 22, 23]. The sympathovagal imbalance may play a crucial part in the pathological mechanism of CKD, as autonomic imbalance leads to lack of nocturnal dip in blood pressure, and diurnal postural hypotension causes hemodynamic changes and endothelial dysfunction. Collectively, these can lead to injury of the glomerular membrane, leading to albuminuria, and thus, a lowering in GFR. Secondly, erythropoietin and anemia may be involved in the association between CAN and CKD, since CAN is related to early dysregulation of erythropoietin production and erythropoietin deficiency anemia. Erythropoietin has a nephroprotective role. Therefore, anemia may be related to eGFR, especially among patients with T2DM.

Most of the risk groups in our study had similar HbA1c levels. This pattern is different from many other studies that had reported that impaired glycemic control contributes to microvascular complications [24, 25]. In a further Spearman's correlation analysis, we found that the relationship between some HRV parameters and kidney function was weaker after adjusting for HbA1c levels. These include the following: LF and LF/HF associations with UACR, LF/HF with eGFR, and SDNN, SDANN, or SDNN index with CKD. This situation is similar to a previous study regarding cardiac autonomic dysfunction and type 1 diabetes mellitus [8]. In that study, the lower and upper UACR groups had significant different HRV parameters but similar HbA1c. The relationship between UACR and HRV parameters, LF and LF/HF, were weakened after adjustment for HbA1c. The result in our study suggests that in T2DM, blood glucose levels may contribute to an association between some parameters of HRV and CKD.

A previous study of Chinese T2DM patients showed that DR was closely associated with both eGFR and UACR [26]. However, in the present study, we found that DR was related to UACR, but not eGFR. Two factors may have contributed to this difference in the results. Firstly, the prevalence of low eGFR (our study 13% compared to previous study 9.94%) and high UACR (our study 38.4% compared to previous study 3.82%), and the cut-off point for UACR (our study UACR ≥ 30 mg/g Cr, previous study UACR > 17 for males and UACR > 25 for females) are different in our study from the previous ones. The prevalence of CKD in our cohort was 37.3%, which is similar to that reported by the Chinese Diabetes Society [15]. This implies that our study sample is truly representative of the Chinese T2DM population. Secondly, the adjustment factors were quite different between the two studies. Our study included additional factors (e.g., BMI, drug history, and concomitant disease) that the previous study did not, which may have affected the association between CKD and DR.

Although we found that BMI was independently associated with eGFR, we did not find a similar result in the regression analysis of UACR. This is inconsistent with a previous research [27]. In our study, the association between BMI and UACR was lost when confound factors entered in the regression equation (aside from age, sex, blood pressure and diabetes status that mentioned in the previous study, we added more that described above). That means different adjustment factors may affect the relationship between BMI and UACR.

In our study, we found age was closely associated with eGFR. However, no correlation between age and UACR was found in our study. This result was supported by a previous study that carried out among 47,204 Chinese adults for the China National Survey of Chronic Kidney Disease [28]. A previous Chinese research showed that other age-related factors such as age at diagnosis of T2DM other than age itself was strongly associated with albuminuria due to the unhealthy lifestyles and genetic factors [29]. Unfortunately, this risk factor was not included in our analysis, but these previous studies might partly explain our result.

The present studied is limited by its cross-sectional design; we could not prove causation, and we studied only associations. Secondly, the subjects of the study population were mainly from the local Yunnan province and may not represent all Chinese ethnicities. In addition, although we recorded the prevalence of hypertension, we missed the exact blood pressure readings of the patients. Since it has been reported that blood pressure is involved in the mechanism underlying the association between HRV and nephropathy [11], we may have learnt more about the association between HRV and CKD if the readings had been known. Finally, we did not record details related to diet, such as dietary salt and magnesium, nor the effect of change of diet on the incidence of hypoglycemic attacks and blood pressure levels.

## 5. Conclusion

In conclusion, our results show that a lower 24-hour time domain HRV parameter, SDANN, was associated with both eGFR and UACR in T2DM Chinese patients. This finding may supply understandings for the physiopathological mechanisms connecting early CAN to increased morbidity and mortality in CKD. Further prospective studies should investigate further these mechanisms and causal associations to explore new treatment strategies for CKD.

## Figures and Tables

**Table 1:** Clinical characteristics of patients according to eGFR and UACR status^a^.

	Low-eGFR^b^	High-eGFR^c^	*P*	UACR_1_^d^	UACR_2_^e^	UACR_3_^f^	*P*
Subjects, *n*	50	334	—	242	72	30	—
Age (y)	67.80 ± 9.84	57.77 ± 11.23	≤0.001	59.06 ± 11.88	58.78 ± 11.21	62.27 ± 8.44	0.325
Female (%)	60.00	52.09	0.296	54.54	55.56	40.00	0.296
BMI (kg/m^2^)	26.80 ± 3.49	24.60 ± 2.96	0.003	24.37 ± 2.73	25.35 ± 3.02^g^	26.11 ± 3.31^g^	0.001
Smoking (%)	4.16	12.10	0.105	11.46	13.79	9.09	0.891
Drinking (%)	4.16	9.76	0.212	10.42	14.29	0	0.17
Diabetes (y)	8 (4-13)	3 (0.16-8)	≤0.001	4 (0.32-8)	8 (2-13.5)^g^	7 (2-20)^g^	0.005
Hypertension (%)	84	52.72	≤0.001	52.5	63.89	73.33 ^g^	0.036
Hypoglycemia (%)	36	17.37	0.002	17.36	33.33^g^	26.67	0.012
Diabetic retinopathy (%)	40	26.50	0.121	19.28	50^g^	66.7^g^	≤0.001
Hemoglobin A1c (%)	8.68 ± 2.60	8.86 ± 2.48	0.648	8.48 ± 2.38	10.16 ± 2.51^g^	8.97 ± 2.58	≤0.001
Blood urea nitrogen (mmol/L)	7.7 (7.0-12.6)	5.1 (4.3-6.3)	≤0.001	5.10 (4.30-6.20)	5.60 (4.45-6.25)	5.45 (4.10-10.60)	0.054
Serum creatinine (*μ*mol/L)	128 (97.8-189.7)	77 (68-89)	≤0.001	80 (69-92)	76.50 (69.50-96.50)	102.25 (96-107)^g, h^	≤0.001
Blood uric acid (*μ*mol/L)	488.93 ± 111.45	342.12 ± 87.57	≤0.001	355.33 ± 102.91	359.15 ± 94.85	427.33 ± 107.90^g, h^	0.019
eGFR (mL/min/1.73 m^2^)	43.64 ± 17.53	87.64 ± 17.45	≤0.001	84.64 ± 21.7	82.19 ± 18.94	59.07 ± 33.18^g^	≤0.001
UACR (mg/g Cr)	33.99 (12.04-591.73)	10.2 (6.41-31.01)	≤0.001	7.86 (5-12.21)	64.57 (35.9-148.58)^g^	1645.06 (1034.1-5057.6)^g, h^	≤0.001
AHT (%)							
Calcium antagonist	36	26.97	0.186	24.37	27.78	40	0.108
RASS inhibitor	36	20	0.011	16.8	27.78^g^	46.67^g^	≤0.001
Beta-blocker	4	6.06	0.561	5.88	8.33	6.67	0.759
Diuretic	12	8.48	0.417	7.56	5.56	20^g, h^	0.042
Diabetes treatment (%)							
OADs	36	41.91	0.428	43.80	36.11	26.67	0.133
Insulin	62	44.91	0.024	48.35	52.78	46.67	0.773

^a^Differences which were analyzed by ANOVA, followed by Tukey's test; ^b^low-eGFR: <60 mL/min/1.73 m^2^; ^c^high-eGFR: ≥60 mL/min/1.73 m^2^; ^d^UACR_1_: <30 mg/g Cr; ^e^UACR_2_: 30-299 mg/g Cr; ^f^ UACR_3_: >300 mg/g Cr; ^g^*P* < 0.05 compared to UACR_1_; ^h^*P* < 0.05 compared to UACR_2_. eGFR: estimated glomerular filtration rate; UACR: urinary albumin : creatinine ratio; BMI: body mass index; AHT: antihypertensive therapy; OAD: oral antihyperglycemic drug.

**Table 2:** HRV parameters in T2DM stratified by eGFR and UACR status.

	Low-eGFR^a^	High-eGFR^b^	*P*	UACR_1_^c^	UACR_2_^d^	UACR_3_^e^	*P*
SDNN (ms)	96 (79.75-134)	121 (98-148)	0.001	123 (103-149)	113 (90-138)^f^	95 (66-110)^f, g^	≤0.001
RMSSD (ms)	40 (23.5-71)	47 (35-72)	0.129	47 (34-76)	46 (33-72)	40 (22-57)^f, g^	0.032
SDANN (ms)	78 (66-114)	117 (89-160)	≤0.001	117 (93-148)	105 (74-132)	74 (66-101)^f, g^	≤0.001
SDNN index (ms)	39 (22-63)	50 (39-62)	0.021	50 (39-62)	50 (35-66)	31 (19-46)^f, g^	≤0.001
LF (Hz)	3072 (256.75-10176)	4356 (651-9050)	0.328	4544 (994-10066)	1320 (468-8332)	593 (110-6701)^f, g^	0.001
HF (Hz)	9568 (422-19664.75)	6639 (862-15988)	0.648	7287.5 (862-19190)	4676 (879-15781)	1383 (125-11749)^f^	0.039
LF/HF (Hz)	0.5 (0.35-0.61)	0.61 (0.47-0.99)	≤0.001	0.57 (0.47-0.98)	0.62 (0.45-0.99)	0.54 (0.43-0.78)	0.606

^a^Low-eGFR: <60 mL/min/1.73 m^2^; ^b^high-eGFR: ≥60 mL/min/1.73 m^2^; ^c^UACR_1_: <30 mg/g Cr; ^d^UACR_2_: 30-299 mg/g Cr; ^e^UACR_3_: >300 mg/g Cr; ^f^*P* < 0.05 compared to UACR_1_; ^g^*P* < 0.05 compared to UACR_2_. eGFR: estimated glomerular filtration rate; UACR: urinary albumin : creatinine ratio; SDNN: standard deviation of the RR interval; RMSSD: the root mean square difference of successive RR intervals; SDANN: standard deviation of the averaged normal RR intervals for all 5-minute segments; SDNN index: the mean of the standard deviations of all normal RR intervals for all 5-minute segments; LF: low frequency; HF: high frequency; LF/HF: the ratio of low-to-high-frequency power.

**Table 3:** Spearman's correlation analysis between different clinical characteristics and HRV analyses.

	SDNN	RMSSD	SDANN	SDNN index	LF	HF	LF/HF
CKD	–0.193^a^	–0.056	–0.223^a^	–0.134^a^	–0.089	–0.019	–0.101
UACR	–0.198^a^	–0.085	–0.176^a^	–0.194^a^	–0.161^a^	–0.093	–0.111^b^
eGFR	–0.012	–0.015	0.074	0.019	0.079	0.013	0.136^a^
Age	–0.047	0.030	–0.165^a^	0.018	–0.04	0.095	–0.241^a^
BMI	–0.129^b^	–0.120^b^	–0.093	–0.111	–0.05	–0.054	–0.008
Diabetes duration	–0.167^a^	–0.123^b^	–0.106^b^	–0.159 ^a^	–0.062	–0.010	–0.122^b^
Hypertension	–0.026	–0.004	–0.092	0.003	0.034	0.051	–0.058
Diabetic retinopathy	–0.166^a^	–0.032	–0.102	–0.142^b^	–0.121^b^	–0.120	0.030
Incidence of hypoglycemia	–0.104^b^	–0.09	–0.055	–0.095	–0.028	–0.039	0.089
Hemoglobin A1c	–0.198^a^	–0.133^b^	–0.041	–0.193^a^	–0.112^b^	–0.108^b^	–0.15
RASS inhibitor	–0.074	0.059	–0.118^b^	0.011	–0.02	0.019	0.058
Diuretic	–0.158^a^	–0.060	–0.150^a^	–0.070	–0.067	–0.045	–0.019
Beta-blocker	–0.093	–0.089	–0.127^b^	–0.102^b^	–0.052	0.014	0.059
Insulin	-0.195^a^	-0.146^a^	-0.128^b^	-0.180^a^	-0.169^a^	-0.129^b^	-0.082
Smoking	0.131^b^	0.071	0.167^a^	0.069	0.104	0.011	0.214^a^
Drinking	0.049	-0.087	-0.02	-0.014	0.039	-0.017	0.140^b^

^a^ *P* < 0.01; ^b^*P* < 0.05. CKD: diabetic kidney disease; UACR: urinary albumin : creatinine ratio; eGFR: estimated glomerular filtration rate; BMI: body mass index; SDNN: standard deviation of the RR interval; RMSSD: the root mean square difference of successive RR intervals; SDANN: standard deviation of the averaged normal RR intervals for all 5-minute segments; SDNN index: the mean of the standard deviations of all normal RR intervals for all 5-minute segments; LF: low frequency; HF: high frequency; LF/HF: the ratio of low-to-high-frequency power.

**Table 4:** Results of binary logistic regression for the independent correlations between renal function and HRV parameters and different clinical characteristics^a^.

	Low eGFR^b^		UACR ^c^	
	Adjusted OR(95% CI)	*P*	Adjusted OR(95% CI)	*P*
SDANN (ms)	0.988 (0.978-0.998)	0.015	0.992 (0.985-0.998)	0.015
Age (y)	1.145 (1.079-1.215)	≤0.001	—	—
BMI (kg/m^2^)	1.209 (1.044-1.401)	0.011	—	—
Diabetic retinopathy (yes or no)	—	—	3.672 (1.844-7.312)	≤0.001

^a^The following were included in both analyses: HRV parameters (LF, HF, LF/HF, SDNN, SDANN, SDNN index, and RMSSD), age, gender, BMI, diabetes duration, drinking status, smoking status, presence of hypertension and diabetic retinopathy, incidence of hypoglycemia, HbA1_C_, insulin, RASS inhibitor, diuretic, and beta-blocker; ^b^eGFR < 60 mL/min/1.73 m^2^; ^c^UACR ≥ 30 mg/g Cr. CI: confidence interval; OR: odds ratio. eGFR: estimated glomerular filtration rate; UACR: urinary albumin : creatinine ratio; SDANN: standard deviation of the averaged normal RR intervals for all 5-minute segments; BMI: body mass index.

## Data Availability

The data used to support the findings of this study are available from the corresponding author upon request.
